RETRACTED

# Efficient lung cancer detection using computational intelligence and ensemble learning

**DOI:** 10.1371/journal.pone.0310882

**Published:** 2024-09-27

**Authors:** Richa Jain, Parminder Singh, Mohamed Abdelkader, Wadii Boulila

**Affiliations:** 1 School of Computer Science and Engineering, Lovely Professional University, Phagwara, Punjab, India; 2 Robotics and Internet-of-Things Laboratory, Prince Sultan University, Riyadh, Saudi Arabia; 3 RIADI Laboratory, National School of Computer Sciences, University of Manouba, Manouba, Tunisia; Jordan University of Science and Technology Faculty of Computer and Information Technology, JORDAN

## Abstract

Lung cancer emerges as a major factor in cancer-related fatalities in the current generation, and it is predicted to continue having a long-term impact. Detecting symptoms early becomes crucial for effective treatment, underscoring innovative therapy’s necessity. Many researchers have conducted extensive work in this area, yet challenges such as high false-positive rates and achieving high accuracy in detection continue to complicate accurate diagnosis. In this research, we aim to develop an ecologically considerate lung cancer therapy prototype model that maximizes resource utilization by leveraging recent advancements in computational intelligence. We also propose an Internet of Medical Things (IoMT)-based, consumer-focused integrated framework to implement the suggested approach, providing patients with appropriate care. Our proposed method employs Logistic Regression, MLP Classifier, Gaussian NB Classifier, and Intelligent Feature Selection using K-Means and Fuzzy Logic to enhance detection procedures in lung cancer dataset. Additionally, ensemble learning is incorporated through a voting classifier. The proposed model’s effectiveness is improved through hyperparameter tuning via grid search. The proposed model’s performance is demonstrated through comparative analysis with existing NB, J48, and SVM approaches, achieving a 98.50% accuracy rate. The efficiency gains from this approach have the potential to save a significant amount of time and cost. This study underscores the potential of computational intelligence and IoMT in developing effective, resource-efficient lung cancer therapies.

## Introduction

Lung cancer is a life-threatening disease that significantly impacts individuals and communities worldwide, leading to severe respiratory complications and a high mortality rate. Early detection is crucial in improving survival rates, making the identification of lung nodules—a potential precursor to lung cancer—a priority in medical diagnostics. With the increasing prevalence of lung nodules, the need for advanced techniques such as Computer-Aided Diagnosis (CAD) systems has become more urgent. These systems, which leverage the power of Computed Tomography (CT) scans, utilize sophisticated X-ray technology to capture images from multiple angles. These images are then processed by computers to generate detailed cross-sectional views of internal anatomy, aiding in the early and accurate detection of lung cancer.

RETRACTED

Early detection of lung cancer is crucial so that effective treatment can be provided to improve the survival rate. Wheezing is the commonly observed symptom of lung-related cancer, which needs special care because of the reason of many individuals who have lung cancer also suffer from a chronic obstructive respiratory disorder, which is the primary cause of coughing. The characteristics behind the cough disease change, which is a critical pulmonary syndrome. Additionally, expectorating, discomfort in the chest, shortness of breathing process, anorexia, weight loss, fever, and bloody sputum are all signs as well as symptoms of lung cancer [1–3].

The conventional diagnostic methods, like X-rays and CT scans, provide detailed images but rely heavily on the expertise of radiologists, leading to potential delays and errors in diagnosis [4–6]. Furthermore, many patients with lung cancer also suffer from chronic obstructive respiratory disorders, which can mask or complicate the diagnosis.

Machine-based learning (ML) techniques and artificial intelligence (AI) approaches are crucial in the healthcare industry. One of the most important applications in healthcare is predictive modeling, which includes developing mathematical models that can predict future outcomes based on existing data [7]. Predictive modeling, for example, can be used to identify individuals who are more likely to develop a particular disease or condition, enabling medical professionals to intervene sooner and treat or prevent the ailment more successfully. Predictive modeling can also be used to improve drug adherence and treatment plans, improving patient outcomes and saving healthcare costs. A variety of laws should be established like in [8, 9] to assess and promote the real-world evolution of software utilities based on AI/ML for the initial presumption and recognition of disease due to the broad application of AI/ML in multiple health disorders’ prediction.

In particular, ML techniques have proved their potential in several healthcare applications [10–14]. Recently, attempts at analyses have also been made to predict different diseases beyond hypertension and diabetes using language models of symptoms [15]. The one that elaborates on how the machine learning domain expanded to include not only the image-based data analysis of skin lesions [16] but also the prediction and management of physiological conditions was further extending an application scope within healthcare [17].

RETRACTED

In this study, many classifiers are compared and analyzed to create a highly sensitive and discrimination-capable model. The benchmark indicators include accuracy, recall, precision, F-Score, and Area Under the Curve (AUC), each crucial component of the diagnostic jigsaw. The proposed method assessments are embellished with AUC ROC curves, which improve the visual comprehension of our models’ effectiveness. In this ever-changing environment, research keeps pace with computational intelligence, where cutting-edge methods like Python-scripted Intelligent Feature Selection, Logistic Regression, MLP Classifier, Gaussian NB Classifier, and a unified Voting Classifier ensemble combine to improve the accuracy of early detection. Computational intelligence and ensemble learning both have their key roles in lung cancer detection, mainly in comparison to techniques developed earlier. Computational intelligence involves using algorithms such as Logistic Regression, MLP Classifier, and Gaussian NB Classifier to improve the analysis of complex datasets, hence greatly improving diagnostic accuracy. Ensemble learning improves this further through methods such as Voting Classifier by fusing several models to avoid false positives. Hyperparameter modification, carried out by diligent grid search, improves model performance further, portending a future in which lung cancer prediction is characterized by accuracy, early action, and lives saved.

The suggested work is an enhanced efficiency and accuracy machine learning-based lung cancer prediction method. This summary outlines the contributions made to this work:

1. This paper introduces a cloud-based IoMT framework for remote patient care, enabling effective data collection, analysis, and sharing with physicians for improved treatment.
2. Logistic Regression, MLP classifier, and Gaussian NB classifier were trained with the dataset. To improve our feature extraction, we combined K-Means clustering with fuzzy logic. We evaluated our model’s performance using accuracy, recall, precision, and F1-score.
3. A voting classifier ensemble with majority voting was used for predictions, and grid search-based hyperparameter tuning was used to boost accuracy and predictive power.
4. Experiments showed the proposed system outperformed current techniques, validating its enhanced performance attaining a remarkable 98.50% accuracy rate.

This study presents an advanced machine learning-based approach for lung cancer prediction, with the following key contributions:

- **Challenge:** Remote monitoring and management of lung cancer patients require an efficient and scalable framework for data handling. **Contribution:** We propose a cloud-based Internet of Medical Things (IoMT) framework that facilitates remote patient care by enabling effective data collection, analysis, and seamless sharing with physicians, thereby improving treatment outcomes.
- **Challenge:** Extracting relevant features from complex lung cancer datasets for accurate prediction is challenging. **Contribution:** We developed a model utilizing Logistic Regression, MLP classifier, and Gaussian NB classifier. To enhance feature extraction, we integrated K-Means clustering with fuzzy logic, leading to improved model performance evaluated through metrics such as accuracy, recall, precision, and F1-score.
- **Challenge:** Single-model predictions often suffer from limitations in accuracy and robustness. **Contribution:** We implemented a voting classifier ensemble with majority voting to combine predictions from multiple models, and further enhanced predictive power through grid search-based hyperparameter tuning.
- **Challenge:** Existing techniques for lung cancer prediction often lack sufficient accuracy and efficiency. **Contribution:** Experimental results demonstrated that our proposed system outperformed existing methods, validating its superior performance and potential for real-world application attaining a remarkable 98.50% accuracy rate.

RETRACTED

The rest of the paper is structured as follows: The relevant existing work is elaborated in the Related Work section, the current approaches are discussed in the Background, and the suggested methodology along with the proposed consumer-focused integrated framework is highlighted in Proposed Methodology. The experimental setup and results of the suggested work are thoroughly detailed and subjected to comparison analysis in Experimental evaluation. The work’s conclusion is presented in the Conclusion section.

## Related work

In this section, we go over the crucial contributions of the researchers in predicting diseases using machine learning models. Nageswaran et al. [18] used machine learning methods and mainly image processing technologies to demonstrate precise classification and anticipation of lung tumors. Gathering photographs was the first step. 83 CT scan images from 70 separate individuals were incorporated into the experimental investigation as the dataset. When processing digital images, the geometric mean filter was employed. Due to this, picture sharpness was improved. The k-mean method was used for the segmentation of photos. After that, machine learning-assisted organizing techniques were applied. It was identified that the ANN architecture is more successful in the prognosis of lung carcinoma.

RETRACTED

Durga V. et al. [19] enveloped a data-driven process and image processing method mainly based on evolutionary techniques for sorting and uncovering breast cancer. To contribute to the segmentation and pinpointing of skin-related chaos, this paradigm integrated image optimization and trait extraction methods. The exponential mean image filter was put into practice to improve the resolution of the scan images. AlexNet was used to extract the features. An algorithm known as relief was used to pick attributes. The proposed architecture used methods such as KNN and Nave Bayes to categorize illness conditions and their identification. Next, data from MIAS was gathered for scientific research. After that, the analysis by using images to accurately diagnose cancer of the breast proved beneficial for the suggested method. Chaudhury S. et al. [20] discussed the framework created for breast-related cancer. An assortment of mammography images was utilized for this framework. To enhance the photos’ holistic quality, the method used is known as contrast-limited adaptive histogram equalization (CLAHE). It’s an improvement upon the traditional histogram equalization technique called CLAHE. In addition to enhancing picture quality, this helps remove noise from pictures. The framework’s development will now move on to picture segmentation. As a result of labeling the pixels at this stage, an image is now separated into discrete sections. This aids in the demarcation of borders and the identification of items. Tactics such as fuzzy-based SVM, Bayesian named classifier, and RF were used, among others, to categorize these pre-processed pictures. Halder and Kumar [21] proposed a unique active learning approach employing a rough-fuzzy classifier (ALRFC) for categorizing cancer disease samples by using gene expression data. The suggested method can deal with overlapping, indiscernibility, and ambiguity of gene expression data. The recommended algorithm was tested using different available illness datasets. The experimental findings for cancer prediction are superior to other cutting-edge methods. According to Chopra et al. [22], the conventional ANFIS is inappropriate for intricate activities of humans, which call for adept manipulation of instruments and systems. The deployment of ANFIS in the progressing domain was explored. The primary ANFIS model was shown to be greatly improved by using metaheuristic approaches and further regulated by nature-inspired algorithms via calibration and adjustment of parameters. It is important for modifying and automating complicated technical activities, particularly in the mechanical, electrical, and geological areas, that now rely on human judgment. The primary purpose of the recommended strategy by Wang J et al. [23] was to investigate the computed tomography (CT) results of pediatric suffered patients who have MPP as well as MP. It is quite frequent, and pediatric respiratory doctors should do crucial studies on treating this type of mixed pneumonia disorder. Raoof et al. [24] used a lung cancer dataset and employed identification of model depending on SVMs. Multiple criteria were used to determine the SVM model’s efficacy. The examined model was inspected using various cancer datasets from the University of California. Sustainable cities will be skilled in providing their residents with improved healthcare due to the positive research findings.

RETRACTED

Kumar et al. [25] discussed the current causes of lung cancer and the usage of ML algorithms, paying particular emphasis to their respective advantages and disadvantages. Instead of referring to several articles, this one allowed the researchers to swiftly scan the pertinent literature. Dritsas and Trigka [26] developed effective models to detect patients who are at high risk of developing lung tumors or cancer and must be treated sooner to avoid long-life consequences. The Rotation Forest was the main approach of the article. In further detail, the trials’ assessment revealed that the suggested model outperformed others with high F-measure, precision, recall, and accuracy. Rajasekar et al. [27] suggested technique exhibits improved performance in the measures. Based on histopathology and CT scan pictures, the suggested method was examined. When histopathological tissues were considered for analysis, the outcome analysis demonstrated that the detection accuracy was higher.

Deepapriya et al. [28] tested several models using a chest X-ray or a CT-scanned image to identify a specific condition. The goal was to determine which deep learning methods best predicted lung illness. Various performance criteria, including accuracy, recall, precision, and Jaccard index, were used to assess the method’s effectiveness. Doyle et al. [29] described the primary diagnosis characteristics of NTMLD patients in the primary care wards and to see if machine learning might be used to recognize NTMLD patients who have not yet received a diagnosis. The UK’s electronic-based medical records primary care database, IQVIA Medical Research Data (a Cegedim Database), was used. Patients with NTMLD were located between 2003 and 2017 based on records of their NTMLD treatment plan or main or secondary care diagnoses. Risk factors and therapies were identified during the pre-diagnosis stage using literature and professional clinical advice. At least one of these traits was added to the control population.112 784 control subjects and 741 NTMLD patients were chosen. From 2006 to 2016, the annual prevalence rates of NTMLD grew from 2.7 to 5.1 per 100,000. For NTMLD patients, COPD and bronchial disorder were the most prevalent pre-existing diagnoses, along with penicillin, macrolides, and inhaled corticosteroids. With an AUC of 0.94, machine learning significantly increased the identification of NTMLD patients compared to random testing. In 2016, it was predicted that there were 9 to 16 diagnosed and unrecognized instances of NTMLD for every 100,000 people. The findings of this study suggest that there may be a sizable number of unconfirmed instances of NTMLD in the UK, supporting the viability of computational learning practiced to primary health data to screen for unverified NTMLD patients.

RETRACTED

Goyal and Singh [30] suggested a unique pattern for predicting respiratory diseases from patient chest X-ray films. The model included feature extraction, responsive and accurate area of interest (ROI) estimate, dataset acquisition, picture quality enhancement, and illness prediction. The researchers utilized two datasets of chest X-ray images that are freely accessible to acquire the datasets. As the picture quality declined while capturing the X-ray, histogram equalization was used to improve it using median filtering. A modified region growth approach that uses dynamic area selection based on resolution intensity degrees and morphological procedures was developed for accurate ROI extraction of chest regions. A strong set of characteristics is essential for the accurate diagnosis of illnesses. From each ROI image, researchers extracted visual, shape, texture, and intensity information before normalizing. A robust normalization strategy was created to enhance detection and classification results. Artificial neural networks, ensemble classifiers, deep learning classifiers, and other soft computing approaches were suggested as a deep learning architecture for accurately diagnosing lung illness. Comparing the suggested model to the current state-of-the-art approaches, experimental findings demonstrate the resilience and effectiveness of the model. The best feature extraction methods were employed by Asuntha and Srinivasan [31]. The Fuzzy Particle Swarm Optimisation (FPSO) method was selected for optimal feature, geometric, volumetric, and brightness characteristics. Deep learning was then used to organize these characteristics. The complexity of CNN’s computational was decreased by the revolutionary FPSOCNN. Besides, this is a real-time data set from Arthi Scan Hospital, and an added valuation was done. The experimental study of data showed that the new FPSOCNN outperforms existing approaches.

RETRACTED

Almarzouki et al. [32] greatly lessen the perplexity of real-time monitoring and data collecting operations for a healthcare practitioner, resulting in better healthcare management. Raising awareness can aid in the development of important dangers and regulating measures. Along with aiding in mitigating strokes, it also detects high-risk variables. In the coming years, the EEG-based brain-computer interface will have a bright future in preventing DALY. Thakur et al. [33] created several techniques based on gene expression. DNA is transformed into Ribose Nucleic Acid (RNA), which is then transported into proteins through gene expression. This protein can be used for many things, such as creating new cells, treating cancer, and even creating hybrid species. Some gene malformations are also passed along to the next generation since genes transport genetic information from generation to generation. Consequently, it’s necessary to find the malformation. To predict malignant and non-cancerous genes using gene expression data, there are several strategies present in the literature. This is a significant breakthrough in diagnosing the illness and providing a prognosis. Ricciuti et al. [34] aimed to ascertain if alterations in the levels of circulating tumor DNA following the start of first-line pembrolizumab treatment in NSCLC would allow early response expectation before radiological evaluation. Plasma patient samples were analyzed by next-generation sequencing employing improved tagged amplicon and coding sections from 36 genes. The outcomes were linked with an early AF. To determine if real-time blood flow radiography may be used to evaluate pulmonary microcirculation scintigraphy in comparison to predict early postoperative lung function and problems, Hanaoka et al. [35] conducted the study. Spirometer and dynamic perfusion digital radiography were done before, as well as one and three months following radical lung cancer resection. The same cases were then used to validate correlation coefficients between blood flow ratios. The relationship between projected values derived from the blood flow ratio and measured taken values was examined for all patients with dynamic perfusion digital radiography.

Lakshmanaprabu, S. K., et al. [36] proposed a new method for the automated diagnosis of lung cancer using CT images. To categorize the nodule in CT lung images as benign or malignant, researchers used the optimal deep neural network and linear discriminant analysis, or in other words, the features have been extracted from the CT lung images through deep transformation and dimensionality reduction. Then, the optimized ODNN has been reached using M-GSA sensitivity, specificity, and accuracy declared as 96.2%, 94.2%, and 94.56%, respectively—one best outcome that confirms the use of an optimized deep learning model for accurate lung cancer classification from CT imaging. This kind of automation can help screen for lung cancer effectively and reliably, allowing radiologists to raise the rate of early detection to improve survival. Althubiti, Sara A., et al. [37] introduced an effective approach for automated lung cancer diagnosis on CT scans. The median filter was the best filter to be applied to medical CT images, which gave better results than the Gaussian, 2D convolution, and mean filters. The preprocessed image was optimized by two optimization algorithms, such as fuzzy c-means and k-means clustering, and later compared. From the two, fuzzy c-means had 98% accuracy. Features of a texture were extracted using the Gray Level Co-occurrence Matrix (GLCM), and three classification algorithms were compared—bagging, gradient boosting, and ensemble, including SVM, MLPNN, DT, logistic regression, and KNN. The best one from this selection was gradient boosting with 90.9% accuracy.

RETRACTED

Table 1 summarizes various studies on cancer detection techniques, comparing methods like ANN, KNN, SVM, and others, using diverse datasets, with observations on the performance and accuracy of each approach.

**Table 1:** Summary of the relevant literature.

Author	Technique Used	Dataset Information	Observations
Nageswaran S, et al. [18]	Artificial Neural Network (ANN), K-nearest neighbor (KNN), and RF	The experimental investigation used a dataset of 83 CT pictures from 70 individual patients.	The results indicate that the ANN outperformed other machine learning techniques in terms of accuracy for lung cancer detection.
V. Durga Prasad Jasti, et al. [19]	Geometric mean filter, AlexNet, Relief algorithm, KNN, LS-SVM, NB, and Random Forest	The study used the MIAS database of 322 mammograms from 161 patients, including various case types, to advance breast cancer detection via image analysis.	LS-SVM achieved the highest accuracy, while KNN exhibited superior sensitivity and specificity for breast disease detection with feature selection.
Wang J, et al. [23]	Chest computed tomography (CT) imaging with MPP and mixed infections of MPP and streptococcal pneumonia (SP). MATLAB is used for analysis.	The pediatric patients’ chest CT scans from the MPP group	Research reveal that chest CT scans differ significantly between children with MPP alone and those with MPP and SP co-infections. The MPP group showed more lung abnormalities and enlarged lymph nodes, while pleural effusions were more common in children with both infections.
C. Anil Kumar, et al. [25]	Support Vector Machine (SVM) classifier for lung cancer prediction, involving data pre-processing, training, testing, feature extraction, and classification.	The study used the Lung Cancer dataset from the University of California, Irvine, which consists of 32 instances, 57 features, and a class attribute.	The SVM classifier, particularly when combined with SMOTE resampling, showed superior accuracy, precision, recall, and F1-score, significantly outperforming other methods such as neural networks and decision trees.
Dritsas, E.; Trigka, M. [26]	Naive Bayes, Bayesian Network, Stochastic Gradient Descent, SVM, Logistic Regression, ANN, KNN, Decision Trees, Random Forest, Rotation Forest, RepTree, and AdaBoostM1.	The research utilized a dataset of 309 participants and 15 features, such as demographic and health-related factors, to predict lung cancer risk.	The Rotation Forest (RotF) model outperformed others with an accuracy of 97.1%, precision, recall, and F-Measure of 97.1%.
Vani Rajasekar, et al. [27]	Inception V3, CNN, CNN GD, Resnet-50, VGG-16, and VGG-19	A dataset comprising CT scan images and histopathological images of lung cancer patients	The CNN GD model achieved the highest accuracy of 97.86%, with a precision of 96.39% and a sensitivity rate of 96.79%.
Deepapriya, B.S., Kumar, P., Nandakumar, G., et al. [28]	Deep learning technique—MSD-NET.	The study focused on predicting lung cancer through deep learning, analyzing chest X-rays and CT scans. Various deep learning models were tested, and their effectiveness was measured by different parameters.	The MSD-NET model demonstrated superior performance to other experimental analysis models.
Goyal, S., Singh. R [30]	ANN, SVM, KNN, RNN, and LSTM	The study utilizes publicly available datasets, C19RD and CXIP, for lung disease detection from chest X-ray images for COVID-19 and pneumonia classification	The F-RNN-LSTM model achieved a detection accuracy of approximately 95%, with significantly reduced computational efforts compared to existing methods.
Hanaoka, J., Yoden, M., Hayashi, K., et al. [35]	Dynamic Perfusion Digital Radiography, Pulmonary Perfusion Scintigraphy, and Spirometry	52 people in total who met the requirements for inclusion were included in the study; however, precise information regarding the dataset was not disclosed.	Dynamic perfusion digital radiography effectively matched with scintigraphy and spirometry, offering a cost-effective method for predicting post-surgical respiratory risks.

RETRACTED

## Background

### The basic classification model

The stages of creating a basic classification model are shown in Fig 1. First, gather and prepare the dataset. Next, clean and preprocess the data for outliers and missing values. Lastly, execute feature selection. Then, divide the dataset into two subsets: training and testing. Select the classification algorithm that fits the problem. Fine-tune the model’s hyperparameters to optimize its performance and evaluate its performance.

**Fig 1:** Generic steps for the classification.

The fact that lung cancer is the primary concern of the demise caused by cancer calls for novel approaches to early diagnosis and treatment. This work uses computational intelligence to develop an environmentally friendly lung cancer treatment model prototype. This strategy promises significant time and money savings through resource optimization and job simplification. A key component of our approach is an intelligent feature selection technique that applies K-Means and fuzzy logic to identify pertinent properties from large datasets on lung cancer. As a result, patient categorization based on symptomatology is more accurate. The Python programming language effortlessly incorporates these procedures by utilizing a variety of classifiers, such as Logistic Regression, MLP Classifier, and Gaussian NB Classifier, and supplemented by a Voting Classifier ensemble framework. Our model’s performance is improved through careful hyperparameter tweaking with the grid search approach, maximizing accuracy and predictive power. This research aims to transform lung cancer detection and therapy by integrating computational intelligence with environmental responsibility. The objective is to increase precision, efficacy, and cost-effectiveness to lessen the effects of this illness on patients and healthcare systems.

### Gaussian Naive Bayes (GNB) classifier

An effective machine learning method for situations where features have continuous distributions is the GNB classifier. The Gaussian (normal) distribution assumption is included in the GNB method, which builds on the Naive Bayes framework. It uses the Bayes theorem to compute posterior probabilities, as shown by Eq (1):

$$\begin{array}{c} P\left(C_{k}|x\right)=\frac{P\left(x|C_{k}\right)P\left(C_{k}\right)}{P(x)} \end{array}$$ (1)

In Eq (1), *P*(*C*_*k*_|*x*) represents the posterior probability, which is the probability of class *C*_*k*_ given the observation *x*. The term *P*(*x*|*C*_*k*_) is the likelihood, which is the probability of observing *x* given that the class is *C*_*k*_. *P*(*C*_*k*_) is the prior probability of class *C*_*k*_, and *P*(*x*) is the marginal likelihood, which is the overall probability of observing *x* across all possible classes. The Gaussian Naive Bayes (GNB) classifier assumes feature independence and a Gaussian distribution for each feature, making it suitable for classifying continuous data.

RETRACTED

### Logistic regression

In machine learning, logistic regression is regarded as a fundamental method that excels at binary classification tasks due to its deceptively straightforward nature. It converts linear combinations into probabilities, denoted by modeling the association between input characteristics and a binary result using the logistic function.

$$\begin{array}{c} P\left(y=1|x\right)=\frac{1}{1+e^{-z}} \end{array}$$ (2)

Here, *P*(*y* = 1|*x*), is the likelihood of the positive class given input x, where z represents the linear combination of the features and weights. Logistic regression is a flexible and well-liked classification method since it identifies subtle patterns in data through repeated optimization.

### MLP classifier

The Multilayer Perceptron (MLP) classifier is a key machine learning component recognized for its capacity to tackle challenging and non-linear classification tasks. An MLP consists of several layers and functions as a neural network. A weighted sum of inputs processed via an activation function, denoted mathematically, determines the output of an MLP node.

$$\begin{array}{c} y=\sigma (w.x+b) \end{array}$$ (3)

Here, y stands for the node’s output for the activation function, w for weights, x for inputs, and b for the bias term. The MLP is a flexible and effective technique for contemporary classification problems because it can capture deep relationships within data through these linked nodes and hidden layers.

### Voting classifier from ensemble learning

Due to its ability to improve prediction performance by mixing many models, ensemble learning has emerged as a fundamental machine learning component. To arrive at a judgment, the Voting Classifier, a well-known ensemble approach, combines the predictions of many classifiers. It uses majority voting for categorization jobs, which is spelled out as follows:

$$\begin{array}{c} y=mode(y_{1},y_{2},\ldots ,y_{n}) \end{array}$$ (4)

Here, y is the final projected class label, but the individual predictions are *y*_1_, *y*_2_, …, *y*_*n*_. The Voting Classifier offers “hard” and “soft” voting algorithms that involve equal collaboration across many models or the averaging of probabilistic predictions for the best possible decision-making.

## Proposed methodology

The suggested method’s flow diagram, shown in Fig 2, includes the following steps:

**Fig 2:** Flow diagram of the proposed methodology.

### Data acquisition

The University of California, Irvine provided the dataset used for this study [38]. The dataset is housed in the Lung Cancer repository, which indicates the database in which the dataset is stored. The UCI lung cancer dataset is a well-known dataset widely used for benchmarking various machine learning algorithms. It serves as the basis of our analysis and consists of 32 instances referred to as individual samples in the dataset. In addition to this, the dataset has 56 characteristics. These refer to the attributes or variables that describe each instance. The dataset comprises many features, including age, gender, alcohol use, genetic risk, chronic lung disease, balanced diet, obesity, smoking, passive smoking, chest pain, blood cough, weight loss, shortness of breath, difficulty swallowing, snoring, and others. [39] Moreover, the dataset contains a single class attribute used in machine learning and data analysis tasks. The class attribute is used to predict or classify the network output.

RETRACTED

### Data pre-processing

In the data pre-processing phase of our study, we imported the lung cancer dataset into Python utilizing the Pandas module. This initial step facilitated data accessibility for subsequent processing steps. To ensure data quality and relevance, we conducted gap-filling and removing irrelevant data. Handling missing values effectively and eliminating superfluous information were essential to maintain the dataset’s integrity and suitability for analysis; Hence, the missing values were dropped. Furthermore, the Synthetic Minority over-sampling Technique (SMOTE) was employed to mitigate any possible class imbalance in the dataset. This technique allowed us to balance the representation of different classes, a crucial consideration in many classification tasks, particularly when dealing with imbalanced datasets. Moreover, to augment our dataset and expand its diversity, we employed synthetic data augmentation technique. These techniques leveraged random functions to generate additional data points, enhancing the dataset’s richness and potentially improving the robustness of our subsequent analyses and machine-learning models. Finally, the normalization is performed using the standardization technique. This approach involves transforming the data with a mean of zero and a standard deviation of one. These comprehensive data pre-processing steps laid the foundation for more accurate and meaningful insights in our study of lung cancer diagnosis.

### K-Fuzzy select feature selection technique

Intelligent feature selection plays a pivotal role in our data analysis process, significantly contributing to the quality and effectiveness of our study. To enhance our attribute extraction efforts, we have incorporated a synergistic approach that combines K-Means clustering with fuzzy logic techniques, which is explained using Algorithm 1 below. K-Means clustering is a well-established unsupervised learning algorithm that excels at identifying natural groupings or clusters within the dataset. We aim to pinpoint cluster data points with common characteristics by applying K-Means. This step is instrumental in uncovering pertinent features within the dataset, as it helps us distinguish relevant patterns and relationships among the variables. We leverage fuzzy logic to refine our feature selection process in tandem with K-Means. Fuzzy logic is particularly valuable in this context because it considers the relevance level associated with each feature. Instead of treating features as strictly binary (relevant or irrelevant), fuzzy logic allows us to assign degrees of relevance, recognizing that some attributes may contribute more significantly to the analysis than others. This nuanced approach to feature selection ultimately increases the attributes’ overall discriminating power. Combining K-Means clustering and fuzzy logic makes our feature selection process more sophisticated and data-driven. We identify relevant attributes and consider their varying degrees of importance, resulting in a more precise and robust set of features for our subsequent analysis and modeling. This intelligent feature selection approach enhances the overall quality and depth of insights derived from our study, ultimately advancing our understanding of the underlying factors in our lung cancer diagnosis research.

RETRACTED

**Algorithm 1** K-Fuzzy Select: Algorithm for Intelligent Feature Selection via K-Means and Fuzzy Logic

**Input:** Input dataset *X* of lung disease samples

**Output:** Optimal attributes Optimal_*f*_

**Start**

Get dataset *X*

Normalize the dataset *X* using the equation:

$$\begin{array}{c} X_{n}=\frac{X-X_{\text{mean}}}{X_{\text{std}}} \end{array}$$

where $X_{\text{mean}}=\frac{1}{n}\sum_{i=1}^{n}X$ and $X_{\text{std}}=\frac{1}{n}\sqrt{\sum {\left(X-X_{\text{mean}}\right)}^{2}}$

Apply k-means clustering technique on dataset *X*_*n*_ and get cluster centers.

Predict the cluster labels for each data point in *X*_*n*_, resulting in *cluster*_*labels*

Determine the number of features, *n*, in *X*_*n*_

Initialize *fuzzy*_*scores* as a zero vector of length *n*

**for** *i* ← *number of features* **do**

 **for** *j* ← *number of clusters* **do**

  Calculate *m*_*s*_ membership value for data in feature *i* with respect to cluster *j* using a Gaussian membership function:

$$\begin{array}{c} X_{\text{mean}}\left(x;c,X_{\text{std}}\right)=e^{-\frac{{\left(x-c\right)}^{2}}{2{X_{\text{std}}}^{2}}} \end{array}$$

where *x* represents the data point values for the *i*-th feature, *c* is the cluster center for the *j*-th cluster and the *i*-th feature

  Calculate *f*_*s*_ fuzzy score using *m*_*s*_ membership value and *c*:

$$\begin{array}{c} f_{s}\left[i\right]=f_{s}\left[i\right]+(\sum_{x\in X_{i}}X_{\text{mean}}\left(x;c_{j},X_{\text{std}}\right))\cdot c_{j,i} \end{array}$$

where *X*_mean_(*x*; *c*_*j*_, *X*_std_) represents the Gaussian membership function for a data point *x* in feature *i*, with *c*_*j*_ being the center of cluster *j* for feature *i*

Get Optimal_*f*_ optimal attributes by finding indices where *f*_*s*_ > 0

**End**

RETRACTED

## Explanation of algorithm steps

- **Normalization:** This step standardizes the input dataset *X* to ensure that all features have a comparable scale. It calculates the mean (*X*_mean_) and standard deviation (*X*_std_) of the dataset and then subtracts the mean from each data point and divides by the standard deviation. Scaling the data yields a mean of 0 and a standard deviation of 1.
- **K-Means Clustering:** The algorithm applies the K-Means clustering technique to the normalized dataset *X*_*n*_. K-Means identifies clusters in the data and computes cluster centers (*c*). Each cluster center represents a group of similar data points.
- **Feature Loop:** The algorithm enters a loop to evaluate each feature in the dataset. This loop iterates through all features, one at a time (*i*), to determine their importance for feature selection.
- **Cluster Loop:** Within the feature loop, there is another loop that iterates through the clusters (*j*). For each feature, this loop calculates membership values (*m*_*s*_) and fuzzy scores (*f*_*s*_) for that feature in each cluster.
- **Membership Calculation (*m*_*s*_):** For each feature (*i*) and each cluster (*j*), the algorithm calculates a membership value (*m*_*s*_) using fuzzy logic. Fuzzy logic allows for a degree of membership rather than a binary classification. It quantifies how well each data point (feature) belongs to each cluster.
- **Fuzzy Score Calculation (*f*_*s*_):** After determining the membership values (*m*_*s*_), the algorithm computes a fuzzy score (*f*_*s*_) for each feature in each cluster. The fuzzy score takes into account the membership value and the cluster center (*c*). This score reflects the importance or relevance of the feature within that cluster.
- **Optimal Attribute Selection:** After calculating membership values and fuzzy scores for all features in all clusters, the algorithm selects the optimal attributes (Optimal_*f*_) based on these scores. The selection process aims to identify the features that are most relevant to the clustering results.
- **End:** The algorithm concludes after evaluating all features and clusters.

RETRACTED

The *K-Fuzzy Select* algorithm is designed to intelligently select optimal attributes by combining K-Means clustering and fuzzy logic. It assesses the relevance of each feature within different clusters, allowing for a more nuanced and data-driven feature selection process. The resulting *Optimal_f* attributes can be used for subsequent analysis, such as building machine learning models or making data-driven decisions in the context of lung disease diagnosis.

### Ensemble voting classifier

**Algorithm 2** Disease Prediction Using Ensemble Voting Classifier and Hyperparameter Tuning

**Require:** Lung Disease Dataset

**Ensure:** Optimized Voting Classifier, Best Hyperparameters, Accuracy Score

1: Get dataset

2: Preprocess dataset

3: Apply feature selection using K-Fuzzy Select algorithm

4: Split dataset into training and testing sets (*X*_tr_, *Y*_tr_, *X*_tt_, *Y*_tt_)

5: Initialize base models for the ensemble: *GNB* ← GaussianNB(), *LR* ← LogisticRegression(), *MLP* ← MLPClassifier()

6: Configure the Voting Classifier with soft voting: *voting*_*clf* ← VotingClassifier(estimators=[(’LR’, *LR*), (’MLP’, *MLP*), (’GNB ’, *GNB*)], voting=’soft’)

7: Define the hyperparameter search space: *H* ← {′*LR*__*C*′: [0.1, 1, 10], ′*MLP*__*hidden*_*layer*_*sizes*′: [(10,), (50,), (100,)]}

8: Initialize and configure GridSearchCV: *GS* ← GridSearchCV(estimator = *voting*_*clf*, param_grid = *H*, cv = 5, scoring = ′*accuracy*′)

9: Perform hyperparameter tuning with GridSearchCV: *GS*.fit(*X*_tr_, *Y*_tr_)

10: Extract the best model and its hyperparameters: M* ← *GS*.best_estimator_, H* ← *GS*.best_params_

11: Evaluate M* on the testing set to measure performance: *Y*_pred_ ← M*.predict(*X*_tt_), P* ← EvaluatePerformance(*Y*_tt_, *Y*_pred_)

12: **return** M*, H*, P*

Our comprehensive classification approach incorporates various machine learning classifiers, including Gaussian NB, MLP, and Logistic Regression. The computational intelligence methods employed, like Gaussian NB, MLP, and Logistic regression, have been explained in the Background section. A Voting Classifier framework, which was synergistically included using Python programming, supports this group of classifiers. The voting classifier is one of the simplest stacking ensemble methods. The Voting Classifier used a soft voting mechanism, where each classifier’s prediction is weighted by its confidence level. The ensemble model configured with the respective parameters of the different machine learning classifiers was optimized through GridSearch. The best models taken with this approach capture linear relationships from LR, complex non-linear patterns from MLP, and probabilistic reasoning with independence feature assumptions from GaussianNB. The predictions from these diverse models were aggregated to get a final prediction resulting in increased accuracy than with just a single model. The disease prediction using an ensemble voting classifier and hyperparameter tuning is explained in Algorithm 2 and Table 2 describes the abbreviations used in the algorithm.

RETRACTED

**Table 2:** Abbreviations used in the algorithm.

Abbreviation	Description
*X*_tr_	Training set features
*Y*_tr_	Training set labels
*X*_tt_	Testing set features
*Y*_tt_	Testing set labels
GNB	Gaussian Naive Bayes classifier
LR	Logistic Regression classifier
MLP	Multi-Layer Perceptron classifier
voting_clf	Voting Classifier with soft voting
*H*	Hyperparameter search space
GS	GridSearchCV for hyperparameter tuning
M*	Best model estimator from GridSearchCV
H*	Best hyperparameters from GridSearchCV
*Y*_pred_	Predicted labels for the testing set
P*	Performance evaluation metrics for the model

### Proposed consumer focused integrated model

Internet of Things (IoT) is a computing concept where each device is interconnected through the internet, and one can communicate with others. IoT is widely used in the medical field, where different IoMT devices play significant roles in collecting and sharing patient data across the network. In Fig 3, cloud-based IoMT architecture has been designed where data can be collected, shared, and analyzed accordingly. Different use cases of IoMT devices have been mentioned here, where n is the number of local servers connected with a main cloud server. The framework is designed so that patient data can be collected, extracted, analyzed, and shared with physicians so that they can treat their patients more effectively from a remote distance and the right care can be provided to the patients.

**Fig 3:** Proposed cloud-based IoMT framework.

Data from m patients are collected through IoMT devices and are shared with the nearest local cloud server. An AI module in the local cloud server is responsible for predicting the classified output. The fetched patient data are extracted and classified in the local cloud server using a defined machine learning algorithm and sent to the Dew servers. The data stored in the dew servers are shared with the main cloud servers and local servers of different health organizations so that doctors, nurses, and patients can access the data. The main cloud server is connected to all the local servers and can exchange information across all the servers.

RETRACTED

Different types of IoMT devices are available and used for different applications. Some devices are used in health organizations, and some are portable or wearable to track daily activities and health status. The devices are connected to the internet through a gateway to exchange data through the proper channels. In Fig 3, it can be observed that the IoMT devices are directly connected with the respective local servers through the gateway. Once the data is collected from the patient’s end, it is sent to the local server through the Internet.

The AI module inside the local server receives the data and preprocesses it initially. The preprocessed data are extracted and classified later using ML algorithms, as explained in the above section. The AI module comes with a predictive output shared with the dew servers and further shared with the main cloud server from the dew servers. Different local servers share the predicted data with the main cloud server, where the main cloud server is connected to hospitals, health research labs, or remote dispensaries. The local Dew server is represented in Fig 4, and different ML algorithms are applied to the dataset. The physicians/health specialists can access the data and share the prescribed feedback with the respective user-ends. The data can be accessed from the local servers so that doctors, nurses, or patients can utilize the stored information anytime.

**Fig 4:** Local cloud server module.

With the proposed framework, an intelligent network environment can be designed between users and healthcare professionals so that appropriate treatment can be possible in time from a remote distance. The intelligent AI module can help classify the disease automatically and smartly so that doctors can prescribe medicines and treat them accordingly.

## Experimental evaluation

This section contains the experimental analysis and findings of predicting lung disease.

### Experimental setup

Our computational experiments were conducted using Jupyter Notebooks, an open-source web application. Jupyter provides an interactive environment well-suited for exploratory analysis and data visualization. The Jupyter environment was set up with a Python 3 kernel, and experiments were executed on a machine with an Intel Core i5 processor, 16GB RAM, and an NVIDIA GTX 1080 Ti GPU. The Jupyter Notebook interface was accessed via a local server on the host machine, ensuring a consistent and isolated environment for all experimental runs.

### Training and testing samples

To assess the performance of our machine learning models effectively, we have partitioned the dataset into two distinct subsets: a training sample and a testing sample. This division is a critical step in our study’s methodology, ensuring that our models are both trained and evaluated rigorously. Specifically, we have allocated 80% of the dataset to the training sample. This substantial portion serves as the foundation for our machine-learning algorithms. During the training phase, our models learn from this data, capturing underlying patterns, relationships, and trends that are essential for making accurate predictions or classifications related to lung cancer diagnosis. Conversely, the remaining 20% of the dataset is reserved for the testing sample. This sample is an independent and unseen data set that our models have not encountered during their training. By evaluating the models on this test sample, we can gauge their generalization performance—their ability to make accurate predictions on new, unseen data. This division into training and testing samples helps us assess the model’s ability to make accurate predictions on real-world, previously unseen cases, a critical measure of its effectiveness.

RETRACTED

### Evaluation parameters

The parameters of evaluation that were considered for the performance evaluation of machine learning models include accuracy, precision, recall, and F-Score [40, 41]. With the contribution of the confusion matrix, these desired metrics were evaluated, consisting of elements: True Positive(TP), True Negative(TN), False Positive(FP), and False Negative (FN). Accuracy measures the proportion of correctly predicted instances, including true positives and negatives, against total instances. Precision looks more at the quality of positive predictions. It is the ratio of true positives to the total predicted as positive. Recall, also known as sensitivity or the true positive rate, measures how well a model can detect all instances of interest. The F1 measure is the harmonic average of both precision and recall, thus balancing between these two measures. The formula for all these metrics is given below:

$$\begin{array}{c} \text{Accuracy}=\frac{TP+TN}{TP+TN+FP+FN} \end{array}$$ (5)

$$\begin{array}{c} \text{Precision}=\frac{TP}{TP+FP} \end{array}$$ (6)

$$\begin{array}{c} \text{Recall}=\frac{TP}{TP+FN} \end{array}$$ (7)

$$\begin{array}{c} \text{F1}\;\text{Score}=2\times \frac{\text{Precision}\times \text{Recall}}{\text{Precision}+\text{Recall}} \end{array}$$ (8)

### Results and discussion

In this section, we report the findings from our thorough examination of classification performance, which considered important parameters, including accuracy, F-score, recall, and precision. We successfully demonstrate the sturdiness of our technique by careful comparison with several existing approaches. Our strategy achieves higher accuracy rates while retaining precision and recall values on par with or beyond those of current techniques. Our inquiry includes a thorough analysis of the components that affect how well our technique performs, revealing potential areas for improvement. These findings highlight the potential of our technique to provide improved accuracy and reliability for classification tasks, placing it as an exciting candidate for practical applications.

RETRACTED

Precision, F1-score, Accuracy, and recall were the four key measures we used in our assessment technique mentioned below in Table 3, to analyze the effectiveness of our classification model. By calculating the percentage of samples that were properly identified out of all samples, we could determine our model’s accuracy. The fraction of samples categorized as genuine positive samples among all samples was also considered while precision was calculated. Recall was computed as the ratio of correctly classified positive samples to all positive samples overall, much like classification. The F-score, a comprehensive performance indicator representing the full power of the model’s categorization skills, was constructed using the harmonic mean of accuracy and recall.

**Table 3:** Simulation parameters and values.

Simulation Parameters	Values
Training dataset	80%
Testing dataset	20%
Machine learning Models	LR, MLP, Gaussian NB, Ensembled Voting Classifier
Constant *c* (LR)	0.1 to 10
Hidden layers (MLP)	10 to 100
Best Constant *c* (LR)	10
Best Hidden Layers (MLP)	50
Hyperparameters Tuning Method	Grid Search Method

In Fig 5, the red bar in the graphical depiction, which shows a significant variance in the number of characteristics, shows that there are more than 50 different traits. Our ideal attribute count criteria imply that an attribute count of fewer than 15 is represented by the blue bar, which is preferable for best performance, which is in opposition to this finding. Firty six features were reduced to fifteen features using the proposed feature selection technique, which thus saved processing time.

**Fig 5:** Comparison of attributes.

Table 4 summarizes the values obtained for the validation and test accuracy metrics for different train-test split ratios of the dataset. The highest test accuracy is obtained for the 80:20 train/test split case; the corresponding confusion matrix is presented in Fig 6. The total execution time was 38.92 seconds. Within this period, the fuzzy logic-based feature selection process was completed in 0.50 seconds, while the ensemble model training took significantly longer, with a total duration of 35.54 seconds. The confusion matrix comes from its capacity to graphically represent a classification model’s performance. This matrix makes it easier to understand how well the model predicts outcomes concerning the labels assigned to each class. The confusion matrix shows 74 true negatives (TN) and 123 true positives (TP) in the context of our particular investigation. Impressive, there have been no false positives (FP) and just 3 false negatives (FN). This astoundingly low percentage of misclassification, especially in predicting the positive class, provides a strong defense of the model’s astounding competence and accuracy.

RETRACTED

**Fig 6:** Confusion matrix (20% data reserved for testing).

**Table 4:** Performance of the model with different train/test split ratio.

Train/Test Split ratio	Accuracy	Precision	Recall	F1-Score
70:30	0.9792	0.98	0.978	0.978
80:20	0.9850	0.9761	1.00	0.9879

ROC curve, shown in Fig 7, illustrates how the classification model balances its sensitivity and specificity. The orange line shows the ROC curve, and its AUC value of 0.98 denotes exceptional performance.

**Fig 7:** Receiver Operating Characteristic (ROC) curve of AUC.

Clear differences in the performance measures are visible in Fig 8 when contrasting the classification results of Naive Bayes (NB) and Fuzzy K-Ensemble techniques. The NB method’s recall, accuracy, and precision are 0.77, 0.78, and 0.77, respectively. These results demonstrate the higher classification skills of the Fuzzy K-Ensemble method, demonstrating its potential for increased precision and accuracy in real-world applications.

**Fig 8:** Comparison of fuzzy K-Ensemble performance parameters with NB classifier.

Different performance patterns can be seen in Fig 9 when contrasting the J48 and Fuzzy K-Ensemble classification techniques. J48 yields an accuracy of 0.76, recall of 0.78, precision of 0.77, and F-measure of 0.76. Conversely, Fuzzy K-Ensemble consistently outperforms the other models, achieving 0.9850 accuracy, 0.9761 precision, 1.00 recall, and 0.9879 significant F-measure.

**Fig 9:** Comparison of fuzzy K-Ensemble performance parameters with J48 classifier.

There are noticeable performance patterns when comparing the SVM (Support Vector Machine) and Fuzzy K-Ensemble classification techniques as depicted in Fig 10. The Fuzzy K-Ensemble consistently outperforms the SVM technique in all four of these measures, with values of 0.9850 for accuracy, 0.9761 for precision, 1.00 for recall, and a noteworthy 0.9879 for F-measure. The SVM strategy results in an accuracy, precision, recall, and F-measure of 0.81 and 0.82. These results highlight the Fuzzy K-Ensemble’s strong accuracy performance.

**Fig 10:** Comparison of fuzzy K-Ensemble performance parameters with SVM classifier.

RETRACTED

Table 5 compares the performance of four different machine learning models—NB, J48, SVM, and our proposed model across four parameters: Accuracy, Precision, Recall, and F-measure.

**Table 5:** Comparison of NB, J48, SVM with FuzzyK-Ensemble.

Parameters	NB	J48	SVM	FuzzyK-Ensemble
Accuracy	0.77	0.76	0.81	0.9850
Precision	0.78	0.77	0.82	0.9761
Recall	0.78	0.78	0.82	1.00
F-measure	0.77	0.76	0.81	0.9879

The paired t-test is the statistical method for comparing two related groups. This research has used it to compare the performance metrics of baseline machine learning models and the proposed model over accuracy, precision, recall, and F1-score with J48, SVM, and NB. The results of the paired t-test are shown in Table 6. Paired t-test results indicate that the proposed model performs significantly better for all metrics under investigation than the baseline models represented by J48, SVM, and NB. Indeed, all the p-values are very small and below the common threshold of 0.05. This will provide very strong evidence to prove that the improvements observed are statistically significant and not due to random chance. Therefore, the proposed model is likely to be a superior choice that will offer a more reliable and accurate prediction.

**Table 6:** Paired t-test results for performance metrics.

Metric	p-value
Accuracy	0.0055
Precision	0.0060
Recall	0.0048
F1-Score	0.0055

The comparison of accuracy results between previous studies and the suggested model presents a clear progression in developing and refining machine learning methods for a specific task. This progression is illustrated in Table 7 through the incremental improvements in accuracy percentages, culminating in the suggested model’s superior performance.

**Table 7:** Comparison results of accuracy between previous studies and suggested model.

Authors Name	Methods used	Accuracy (%)
Gultepe Y. [39]	KNN, NB, DT	83
Faisal et al. [42]	Majority voting ensemble model	90
Patra R. [43]	RBF classifier	81.25
Khashei M et al. [44]	DIMLP	94.43
Our Work	Fuzzy K-Ensemble	98.50

The limitation of the model is that it was tested only on lung cancer; however, its generalizability needs to be tested for other types of cancers also. There are no defined measures of the model’s performance concerning accuracy, precision, recall, and F1 score against other cancer types. Different cancers have different characteristics and genetic profiles. A model trained using lung cancer data may not effectively capture the relevant features to predict other cancers.

## Conclusion and future work

To sum up, the fact that lung cancer is a primary cause of cancer-related death highlights the urgent need for novel approaches. This research capitalizes on recent computational intelligence advancements to establish an environmentally conscious prototype for lung cancer treatment, offering optimized resource utilization and potential time and cost savings. Intelligent Feature Selection, Logistic Regression, MLP Classifier, Gaussian NB Classifier, and Voting Classifier ensemble methods, all implemented using Python, collectively enhance early detection accuracy. Hyperparameter tuning through grid search further refines the model. Comparative analysis against existing methods substantiates the proposed model’s superior performance, attaining a remarkable 98.50% accuracy rate. These findings highlight the transformative potential of computational intelligence in advancing effective lung cancer diagnosis and treatment paradigms.

RETRACTED

Given this study’s promising results, several future work directions could be proposed. First, it would further enrich data with additional modalities, like genomic or EHR data, to strengthen predictive power and robustness. Another avenue is using deeper architectures, like Convolutional Neural Networks for image data and Recurrent Neural Networks for sequential data. It can leverage transfer learning with pre-trained models on large medical datasets to improve performance on specific lung cancer datasets.

Another important area would be developing a real-time lung cancer detection system that clinically integrates seamlessly into workflows. Ensuring that such a system is user-friendly for clinicians and providing fast and reliable results is also essential. Further enhancing model accuracy would be exploring new techniques to derive more informative features and using automated tools to discover possible new features.

The next step should be rigorous cross-validation and external validation to ensure generalizability across different subsets. Validating this model on datasets most external to these subsets, originating from different populations and institutes of medicine, will help confirm its robustness and applicability. Such future research directions will guarantee that computational intelligence will reach its full potential for improving the diagnosis and treatment of lung cancer, leading to improved patient outcomes and more efficient healthcare systems.
